# Time Series Anomaly Detection Model Based on Multi-Features

This article has been retracted.

**DOI:** 10.1155/2022/2371549

**Published:** 2022-08-08

**Authors:** Hengyao Tang, Qingdong Wang, Guosong Jiang

**Affiliations:** Computer School of Huanggang Normal University, Huanggang, Hubei 43800, China

## Abstract

For Internet information services, it is very important to closely monitor a large number of key time series data generated by core business for anomaly detection. Although there have been many anomaly detection models in recent years, its practical application is still a big challenge. The model usually needs repeated iteration and parameter adjustment; and for different types of time series data, we need to select different models. Therefore, this paper proposes an anomaly detection model based on time series. The model first designs the statistical features, fitting features, and time-frequency domain features for the time series, and then uses the random forest integration model to automatically select the appropriate features for anomaly classification. In addition, this paper presents an anomaly evaluation index ADC score with timeliness window, which adds the time delay factor of anomaly detection on the basis of F1-score. We use the KPI time series, a representative key performance index in the industry, as the experimental data. It is found that the ADC score of the anomaly detection model in this paper reaches the level of 0.7–0.8, which can meet the needs of practical application.

## 1. Introduction

The purpose of time series anomaly detection is to find data that do not conform to the common rules in time series, that is, abnormal data. Time series anomaly [1–3] refers to that time series data will show some characteristics with a different severity (such as fluctuation), which is an important research content in the field of time series analysis. Outliers usually seriously affect the statistical analysis and prediction of time series.

With the rapid development of the Internet, the scale of information services is growing day by day. In order to ensure uninterrupted business, the operation and maintenance personnel need to closely monitor a large amount of timing data generated by their core business at any time. Therefore, it is more and more important to ensure the stability of its services. The operation and maintenance personnel judge whether the service is stable by monitoring various timing data, because the timing data are abnormal. It often means that there are potential failures in its related application services, such as server failure, network overload, and external attacks. If the corresponding exceptions are not eliminated in time, it is likely to cause damage to its user experience, resulting in a huge economic cost in revenue. Therefore, it has very important research significance in theory and practical application.

In the specific identification of abnormalities, the definition and severity judgment of the operation and maintenance personnel will change with different time series. Because the operation and maintenance personnel usually judge the exceptions according to their understanding of business data and real operation and maintenance needs, these exceptions are difficult to be defined by some preset rules.

In this paper, we assume that the statistical characteristic criteria considered by operation and maintenance personnel in determining exceptions do not change over time. This paper focuses on a kind of time series, which is an abstract service based on the Internet. It monitors and detects the exceptions of KPI (key performance indicator, such as CPU utilization, queries per second, response delay) time series of its applications and systems, so as to maintain the reliability of its services [2, 4–6]. Considering the following reasons in the current actual scene, first, the characteristics of time series in the data set are different, some are periodic, and some are stable and unstable, rather than simple periodicity. Second, the real industrial data set used has a complete label and meets the conditions of supervised algorithm. Third, the current unsupervised learning algorithm is only for periodic time series, and the length of each time series is required to be at least 6 months. At present, the data in the data set are only one month, which is far from meeting its requirements. In this paper, supervised machine learning algorithm is selected for anomaly detection of time series, rather than unsupervised method only for periodic data.

First, the contribution of each training model is different from that of the previous research. We take the time series data with different feature types as a training set to train a general model. This is because in the actual application scenario, the data scale of time series is very large. It is almost impossible to configure and optimize the algorithm parameters for each time series. This requires the algorithm to have sufficient stability and universality, and achieve good results. Second, considering that under normal circumstances, the operation and maintenance personnel often care about whether the anomaly detection algorithm can detect a continuous anomaly interval, rather than detecting each anomaly point in the interval. Therefore, this paper also innovatively proposes an anomaly detection and evaluation method ALC score with timeliness window. For continuous abnormal points, the evaluation method specifies the timeliness window. As long as the abnormal points are detected in the window, the abnormalities in this section are counted as successful detection; otherwise, it is judged as failure. This method improves F1-score formula and is closer to the actual industrial application scenario.

## 2. Related Work

Time series analysis and mining have attracted attention in recent years [7]. Time series applications have been widely used in transportation [8], operation and maintenance [9–11], and medical [12–15] fields. At present, the development status of time series anomaly detection algorithm can be roughly divided into three stages. The first stage is to use traditional statistical algorithms. Statistical algorithms can also be roughly divided into two categories. The first method directly models the time series of normal behavior. When a point has a significant deviation, it is considered an outlier. These methods mainly include ARIMA, exponential smoothing, Kalman filtering, and state space model. The second method is based on the idea of time series decomposition. In time series analysis, the time series is usually divided into three elements: trend, seasonality, and noise. By monitoring the noise component, abnormal values can be captured. This method needs to select a reasonable threshold strategy to judge the outliers.

The second stage is to use supervised machine learning algorithm. Construct the framework and system of anomaly detection based on supervised machine learning. The representative of this stage is Yahoo's EGADS system. For the traditional statistical algorithm anomaly detector, the parameters and threshold of the detector need to be adjusted manually and iteratively. Use detection based on static threshold to solve the problem. The anomaly detection system based on supervised machine learning technology takes the apprentice system as an example. This can capture complex concepts based on the characteristics and labels of the data. The only manual work of the operator is to use convenient tools to regularly mark exceptions in the performance data. Several existing detectors are applied to performance data in parallel to extract abnormal features. Then, features and labels are used to train the random forest classifier to automatically select the appropriate detector—parameter combination and threshold. The apprentice system can automatically meet or approach reasonable accuracy preferences (recall rate is greater than or equal to 0.66, and accuracy rate is greater than or equal to 0.66).

The third stage is to use unsupervised depth generation learning algorithm to solve the challenge of seasonal and unlabeled time series anomaly detection. For large Internet companies, it is necessary to closely monitor various time series KPIs of their web applications (such as page views, number of online users, and number of orders). However, anomaly detection of these seasonal KPIs with various patterns and data quality has always been a great challenge, especially without labels. Therefore, the researchers first proposed an unsupervised anomaly detection algorithm donut based on VAE. Due to the performance of the most advanced apprentice method, VAE-0 is far better than the most advanced apprentice method. A new explanation of KDE reconstruction donut is also proposed, which makes it the first VAE-based anomaly detection algorithm with solid theoretical explanation.

Then, the researchers proposed bagel, an unsupervised time series anomaly detection algorithm based on conditional self-encoder (conditional VAE). The main purpose of this method is to solve that donut is not a sequential model and cannot deal with time-related anomalies. CVAE combines time information and dropout layer to avoid over-fitting. Compared with donut, bagel improved the best F1-score by 0.08 to 0.43.

Of course, in these development stages, there are many other development directions for anomaly detection of time series, such as anomaly detection for concept drift of time series. A typical example is the drift of network traffic. Generally speaking, at a certain characteristic time point, the time series will fall or rise sharply. However, the trend after falling or rising is very similar to the historical data, but the absolute value changes. There are two ideas here. The first is to change point detection. Some propose SST algorithm based on SVD algorithm, which has a certain time complexity. Later, there is robust SST based on SST. The second is the judgment of similarity. From a mathematical point of view, it is to judge whether the two time series are similar. Therefore, some scholars propose to judge whether there is a linear relationship between the old concept and the new concept through the algorithm of linear regression, that is, whether they are only translational.

## 3. Time Series Anomaly Detection Model

### 3.1. Challenges

Although the above supervised machine learning is very expected, it faces many challenges when it is applied to the scene of real time series anomaly detection.

#### 3.1.1. Category Imbalance

In the problem of anomaly detection, the number of normal samples is always much more than that of abnormal samples. Therefore, when the original data set is directly used for model training, the classifier will seriously tilt to the normal samples and ignore a small number of categories. This will lead to the reduction of test results and cannot meet the needs of operation and maintenance personnel. For this problem, we try several schemes: (1) under sampling normal samples to achieve positive and negative samples of 1 : 1; experiments show that this scheme will have serious over-fitting and poor generalization performance due to the loss of a large amount of sample information; (2) oversampling of abnormal samples to achieve 1 : 1 of positive and negative samples. Finally, the decision is adjusted through the threshold. The measured results of this method are ideal, which has become our final scheme.

#### 3.1.2. Irrelevant and Redundant Features

In order to reduce the labor cost, we neither choose the most appropriate feature extraction methods nor adjust their internal parameters. On the contrary, we use many feature extraction methods to obtain features at the same time, some of which may be irrelevant or redundant. Previous work has proved that some learning algorithms will be affected by redundant features, thus reducing the accuracy. We solve this problem by using an integrated algorithm—random forest.

### 3.2. Feature Extraction

This section introduces the eigenvalue extraction methods widely used in time series analysis selected in this paper for time series anomaly detection, which can be divided into three categories: (1) traditional statistical features, (2) fitting features, and (3) time-frequency domain wavelet features. Through these feature extraction methods, different eigenvalues are extracted from the time series, the information of the time series is summarized into this group of eigenvalues, and some considerations in selecting the feature extraction method are introduced.

### 3.3. Statistical Feature

This section will briefly introduce the statistical eigenvalues used in this article and how these eigenvalues are used in this article.

Logarithmic characteristics [16]: In KPI time series, there are many outliers related to zero value. When the relevant data of the system suddenly become zero, there is likely to be an exception. Therefore, in many previous experiments, take the KPI time series data as the right value. Because of the nature of the log function, when the data value tends to zero, the log function value will tend to negative infinity. Through this simple processing method, it can have a significant effect on outlier detection in KPI time series.

Statistical order moment characteristics [17]: Among the various statistical characteristics of KPI time series, the first-order distance to the fourth-order distance are the statistical characteristics often used in previous studies. The four steps are mean, variance, skewness, and kurtosis. Variance is the most important eigenvalue to measure the fluctuation of data, which reflects the dispersion of a group of data. It is the square of the difference between each sample value and the overall average value, which is of great significance to the degree of deviation of the research data. In KPI time series, many abnormal points are characterized by steep rise or fall, that is, deviation from adjacent data. Therefore, the variance measure is very suitable for capturing such outliers. Skewness is a measure of the direction and degree of skewness in the distribution of statistical data. Kurtosis is a measure of the kurtosis of the probability distribution of a group of data. It is the difference between the fourth-order origin moment of any standardized variable and standardized normal variable. Under the same standard deviation, the greater the kurtosis coefficient, the more sharp or extreme the values of the data distribution. Therefore, the four order statistics are used to obtain the concentration, fluctuation, asymmetry, and extreme value of KPI time series.

Difference and difference ratio [18]: Generally, the difference refers to the difference between two adjacent items in the data, while the difference in the KPI time series has a broader meaning. We sampled the difference between the current data point and the adjacent previous point, and the difference between the current data point and the point in the previous day cycle.

### 3.4. Fitting Feature

The greater the distance between the prediction point and the time series, the clearer the prediction point. Suppose that the time change weight decreases exponentially—the most recent is 0.8, then 0.8 *∗* 2, 0.8 *∗* 3, and so on. Finally, the weight of old data is close to 0. The weight is attenuated according to the exponential order, which is the basic idea of exponential smoothing method. In time series anomaly detection, the basic idea of exponential smoothing method is used to predict the current point, and then the difference between the real value of the current point and the predicted value is used as the feature. If the difference is too large, it is likely to indicate that the point is not generated according to the expected pattern and may be an abnormal point. Therefore, we use a variety of different exponential smoothing methods as the fitting features of anomaly detection algorithms.

Primary exponential smoothing [19]: The one-time exponential smoothing method is an adaptive model, which is suitable for the case that the time series value fluctuates randomly up and down a constant mean without trend and seasonality. It is suitable for fitting the time series with unstable characteristics in KPI time series data. Its recurrence relationship is as follows:

(1) $$\begin{array}{c} s_{i}=\alpha \times x_{i}+\left(1-\alpha \right)\times s_{i-1}. \end{array}$$

Quadratic exponential smoothing [20]: The quadratic exponential smoothing method retains the smoothing and trend information, so that the model can predict the time series with trend, and is suitable for fitting the time series with trend in KPI time series data. Quadratic exponential smoothing has two formulas and two parameters. The formula is as follows:

(2) $$\begin{array}{c} s_{i}=\alpha \times x_{i}+\left(1-\alpha \right)\left(s_{i-1}+t_{i-1}\right),\\ t_{i}=\beta \times \left(s_{i}-s_{i-1}\right)+\left(1-\beta \right)t_{i-1}. \end{array}$$

Cubic exponential smoothing [21]: Cubic exponential smoothing, also known as Holt winter method, is a pattern that occurs repeatedly in each fixed time interval, which is commonly referred to as periodicity. This method is suitable for fitting the periodic time series in KPI time series data.

### 3.5. Wavelet Feature

As a signal analysis method, wavelet transform analysis can decompose the time series into low-frequency part and high-frequency part almost losslessly by using the principle of multi-scale analysis. Then, put the decomposed signal into different scales for analysis. It is used as a time-frequency domain analysis method. This method can effectively extract the main information such as random term, periodic term, and trend term. Therefore, it has a good detection effect for the time series with periodicity and trend in KPI time series data. The schematic diagram of wavelet transform decomposition is shown in Figure 1. Taking three-layer decomposition as an example, *T* represents the original time series, A1, A2, and A3 represent the low-frequency parts of layers 1 to 3, and D1, D2, and D3 represent the high-frequency parts of layers 1 to 3. It can be seen from the figure that wavelet decomposition can gradually observe the characteristics of time series from the whole to the details, and it constantly decomposes time series into low-frequency and high-frequency parts. Therefore, it has the characteristics of multi-resolution, which realizes multi-scale analysis.

There are continuous wavelet transform, discrete wavelet transform, orthogonal wavelet transform, and so on, among which the most commonly used is discrete wavelet transform. In practical application, the first problem is to select the appropriate wavelet basis function. This paper selects DB4, coif4, Sym8, dmey, and rbio2 by referring to the previous selection of wavelet transform time basis function of time series and combined with the data characteristics of KPI time series data set 8. For the time series anomaly detection, the high-frequency part decomposed by the information time wavelet transform is mainly used to obtain the abnormal information.

### 3.6. Feature Selection Method

When selecting features, two general conditions need to be met: first, the features need to be suitable for the model, or they can measure the severity of the current data point. In fact, many features can meet this requirement, so this requirement is not high. There are many such features to choose from. Secondly, because anomaly detection needs to meet the needs of timeliness, we require that the detection can be carried out online, which requires that once the data point arrives. Considering the improvement of computer performance, this is not difficult to meet. In addition, some features need a preheated data interval, such as EWMA fitting features. We detect this problem by skipping detection in the preheating interval, which has no impact on predicting future data. Since we hope to release the operation and maintenance personnel from the process of feature selection, we roughly selected the features that meet the above conditions, although there will be redundancy. However, the classification algorithm has great robustness, so there is no need to worry.

## 4. Proposed Model

The time series anomaly detection task in this paper is essentially transformed into a classification problem through supervised machine learning algorithm. At present, there are many commonly used methods for classification problems, such as linear support vector machine. However, due to a large number of redundant and irrelevant features in time series anomaly detection task, considering this, this paper selects the integrated algorithm random forest as the classifier of time series anomaly detection task. Compared with other classification algorithms, this algorithm has the following advantages: (1) less parameters need to be adjusted; (2) it has strong robustness to redundant and irrelevant features; (3) the sensitivity to parameter adjustment is not high. In addition, the characteristic of random forest insensitive to parameters is also very suitable for avoiding repeated adjustment and iteration.

### 4.1. Random Forest Principle

#### 4.1.1. Decision Tree

Random forest is composed of decision tree [22, 23], so let us briefly introduce the concept of decision tree. Decision tree is a basic process of classifying instances based on features. It can be regarded as a set of if then rules, or as a conditional probability distribution defined in feature space and class space. The advantage is that the computational complexity is not high, the output result is easy to understand. But it is prone to over-fitting. Decision tree is a popular learning algorithm because it is easy to understand and interpret [24].

#### 4.1.2. Integrated Learning

Ensemble learning is to complete the learning task by constructing and combining multiple learners, which is sometimes called multi-classifier system [25, 26]. For a single learner (such as decision tree algorithm), if the integration algorithm is homogeneous, then a single learner is called as “basic learner,” and random forest is called as homogeneous integration algorithm. The integration algorithm will obtain better generalization performance than a single learner, especially for “weak learners.” Therefore, in order to obtain the integration with strong generalization ability, we should make a single learner as different as possible. Therefore, in the random forest, we will sample the training samples to produce different subsets and then train a basic learner. In this way, due to different training data, the basic learners we obtain will be greatly different, but in order not to make a single trainer too bad, we use overlapping sample sets. Bagging is a representative of parallel integrated learning algorithm. It is based on self-help sampling method. Given a data set containing *m* samples, we first randomly take out a sample and put it into the sampling set, and then put the sample back into the initial data set. It is still possible to select the next sampling. In this way, after *M* random sampling, we can get the sampling set of *M* samples. Some samples in the training set will appear many times or never appear. Basically, there will be 63.2% of the samples in the sampling set. In this way, we can train *t* basic learners and then combine these learners. This is the process of bagging. Bagging makes a simple voting method for classification tasks. If the number of votes is the same, it will be selected randomly. It can also be determined by further investigating the confidence. If the complexity of the basic learning device is assumed to be *o* (*m*), then the complexity of bagging is roughly *t* (*O* (*m*) + *O* (*s*)). Because the complexity of the sampling and voting process is not high, it can be said to be very small, so *t* is a small constant. Therefore, it shows that bagging integration is of the same order as the complexity of the basic learning algorithm, and it is a very efficient integration method. Random forest is an extension of bagging algorithm. Based on the decision tree as the base learner and the bagging algorithm, random attribute selection is introduced; that is, for each base decision tree, a subset containing *K* attributes is randomly selected from the attribute set of the node, and then an optimal attribute is selected for division. Generally, assuming that there are *d* attributes, *k* = log2d is recommended. Random forest is simple and easy, with low computational overhead, and can be calculated in parallel. It is suitable for large-scale data processing and has strong robustness to redundant features. Based on the above advantages, in the anomaly detection algorithm of time series in this paper, we use random forest algorithm, in which all trees grow repeatedly without pruning operation. By default, the random forest algorithm uses 50% as the classification threshold. In this paper, the classification threshold will be adjusted to obtain the best performance.

### 4.2. Random Forest Application

The implementation of random forest and partial feature extraction algorithm used in this paper is completed by using scikit-learn tool. scikit-learn is an open-source Python machine learning library with many built-in machine learning modules and many data sets. Taking the random forest algorithm as an example, the use steps of scikit-learn tool are as follows:

1. Prepare the data set according to the requirements of scikit-learn toolkit.
2. Clean and scale the data set.
3. Choose which machine learning algorithm to use (random forest in this paper).
4. Cross-validation is used to select the best parameters of random forest—the maximum depth of decision tree and the maximum number of available features.
5. Using the best parameters, the whole training set is trained to obtain the random forest model.
6. The training set and test set are used to test the model, respectively.

The data set used in this paper includes three parts: timestamp, eigenvalue, and exception tag, which are divided by behavior units. The exception tag represents whether data are abnormal. The data set uses 0 and 1 to correspond to normal and exception tags, respectively. In order to avoid the different values of different time series, the values of some time series data are too large and the other part is too small, which leads to unnecessary errors in model training. Therefore, the scaling normalization operation is carried out for each time series. The upper limit of the scaling operation is 1, and the lower limit is 0. Scaling operation can also speed up the training of random forest model and improve the accuracy of the model. Because there are still missing values in the data set, we use the linear interpolation filling method.

## 5. Results and Analysis

This paper adopts six representative KPI data. The time series characteristics include periodic, stable, and unstable. These data are the real data of the industry, from eBay, Tencent, Baidu, and other companies. The labels of data are truly marked by the operation and maintenance personnel, and the abnormal proportion ranges from 0.08%–5.06%. The sampling frequency of the data set is 1 or 5 minutes, and the time span of each time series is 1 month. These data are not only special cases, but also widely representative. There are many data in other fields similar to them, for example, the round-trip time and traffic flow in the field of transportation, as well as the number of online shopping in the field of e-commerce. Therefore, we believe that these six KPI data can reflect the performance and characteristics of random forest algorithm. We also hope to use data and labels in other fields to try our algorithm framework in the future.

### 5.1. Model Results

#### 5.1.1. Evaluating Indicator

Usually, we use error rate and accuracy to measure the quality of the model, but this does not meet the needs of all tasks. For example, in the time series anomaly detection task, the error rate measures the proportion of anomalies that are judged to be wrong, but usually the operation and maintenance personnel are concerned about “how many of the detected anomalies are real anomalies” or “how many of all the real anomalies are detected,” so the error rate is far from enough. Similar requirements often appear in web search and information retrieval tasks, “precision” (P for short), and “recall” (*r* for short), as well as their combination index F1-score. The formula is as follows:

(3) $$\begin{array}{c} P=\frac{\text{T P}}{\text{T P}+\text{F P}},\\ R=\frac{\text{T P}}{\text{T P}+\text{F N}},\\ F1=\frac{\left(2\;\times P\;\times R\right)}{P+R}. \end{array}$$

It is more suitable for such needs. Similarly, these three indicators are also more in line with time series anomaly tasks. Therefore, this paper also uses these three evaluation indicators. However, in the communication with relevant operation and maintenance personnel, it is found that these three indicators do not take into account the requirements for time delay in time series anomaly detection tasks. Therefore, we also innovatively put forward ADC score. This preference score increases the focus on time delay on the basis of F1-score.

#### 5.1.2. Result Evaluation

Joint training can greatly reduce the model training cost in the actual scene. In the actual scene, the operation and maintenance personnel often care about whether the anomaly detection algorithm can detect a continuous anomaly interval under a certain time delay, rather than detecting each anomaly point in the interval. Therefore, we improve the evaluation standard in the joint training model and use ADC score. To make the model more suitable for industrial application scenarios, the ADC score evaluation criteria are as follows: for continuous abnormal points, it is specified that the timeliness window is 7-point interval (i.e., 7 minutes, 35 minutes if the interval is 5 minutes). As long as abnormal points are detected in the window, the abnormalities in this section are counted as successful detection; otherwise, it is judged as failure. For this standard, we added the weight of the first seven points in the abnormal interval during model training, so as to hope the model can learn their importance.  Table 1 shows the performance of the model in accordance with the actual situation.

As can be seen from the table, considering the evaluation standard ADC score of timeliness window, the performance of the algorithm will be greatly improved, basically reaching the level of 0.7–0.8. The robustness of the model to the forest operation and maintenance personnel can basically meet the requirements of this model.  Figure 2 presents the first KPI data PR curve.

### 5.2. Result Analysis

This paper implements a time series anomaly detection algorithm. According to several feature extraction algorithms, a set of features including statistics, fitting, and wavelet are extracted from KPI time series. These characteristics play a great role in time series analysis. The machine learning classification algorithm selected in this paper is random forest, which has fewer parameters. It is insensitive to parameters and has strong robustness to redundant and irrelevant features. For different data sets, it can automatically select the best feature combination among a large number of features. The ADC score evaluation index proposed in this paper creatively combines the requirements of anomaly detection for time delay. The operation and maintenance personnel are concerned about the abnormality in time. Instead of detecting every point in the abnormal interval, thus, the performance of the algorithm in anomaly detection task is greatly improved. It is worth mentioning that in this paper, the selection of features and the sampling of parameters are not very carefully selected, but most of the common and meaningful features in time series analysis are widely selected. Therefore, the performance of the algorithm has further potential.

## 6. Conclusion and Prospect

Based on the real KPI time series data set in industry, this paper uses random forest algorithm to realize the goal of anomaly detection of time series data and selects some important features in time series analysis, including a large amount of time series information in time-frequency domain such as statistics, fitting, and wavelet. The experimental results show that compared with some early research schemes, the ADC score evaluation index with time window is proposed, which is closer to the needs of the real scene of timing anomaly detection, and has achieved good detection results. The joint training of multiple time series is also in line with the common existence of a large number of different types of time series in the real scene, and the random forest algorithm itself is suitable for parallel computing, which also makes the practical application prospect of the algorithm very objective. However, there are still large errors in the algorithm. We hope to further improve the detection results of the algorithm in the future. In addition, for the future, the goal of this paper is to realize automatic machine learning, called automl. Its purpose is to automate the whole process of machine learning and reduce the labor cost in data preprocessing, feature engineering, model selection, and parameter adjustment. The main function of automl is to help more people without professional knowledge to build efficient models and adjust super-parameters. This involves Bayesian optimization, reinforcement learning, migration learning, and so on. The data in some applications can only be obtained in batches, such as daily and weekly, and the data distribution changes relatively slowly over time, which requires automl to have the ability of continuous learning or lifelong learning. In the artificial intelligence top-level conference neurops 2018 and pakdd 2019 automl challenge, we began to pay attention to concept drift, rather than simple independent and identically distributed, which is closer to reality. Most of the problem data in the real-world are different, while the previous automatic machine learning framework only supports numerical types. The participating team designed to extend automatic machine learning to a variety of data types and introduced different types of feature preprocessing and feature engineering and feature combination of different types of features, so that automl can be applied to more real-world problems without expert intervention. There is often concept drift between real data, and there are a large number of category imbalance problems. The model needs repeated training to adapt to concept drift, and experts need to deal with concept drift and category imbalance. The framework designed by our team adapts to the concept drift by integrating the data of different periods and combining the training of DNN and lightgbm, introduces adaptive sampling, and improves the sampling rate of gradient lifting model to alleviate the category imbalance and realize lifelong machine learning. The lifelong automated machine learning framework can be applied to various real-world problems, such as anomaly detection, recommendation system, online advertising, fraud detection, transportation monitoring, econometrics, patient monitoring, and many other fields. Without the intervention of domain experts, our framework can train a model with high performance, strong timeliness, and feasible time, so as to reduce the application threshold, shorten the project development cycle, and promote the large-scale implementation of machine learning.

## Figures and Tables

**Figure 1:** Schematic diagram of wavelet transform decomposition.

**Figure 2:** Case study. The first KPI data PR curve.

**Table 1:** The performance of the model in accordance with the actual situation.

	0th	1th	2th	3th	4th	5th
F1-score	0.48	0.14	0.58	0.68	0.54	0.62
ADC score	0.68↑	0.72↑	0.72↑	0.83↑	0.76↑	0.82↑

## Data Availability

The data set can be accessed upon request.

## References

[1] Teng M. Anomaly detection on time series.

[2] Ren H., Xu B., Wang Y. Time-series anomaly detection service at microsoft.

[3] Salvador S., Chan P., Brodie J. Learning States and Rules for Time Series Anomaly Detection.

[4] Qiu J., Du Q., Qian C. (2019). KPI-TSAD: a time-series anomaly detector for KPI monitoring in cloud applications. *Symmetry*.

[5] Wang C., Wu K., Zhou T. (2021). TSAGen: Synthetic Time Series Generation for KPI Anomaly Detection. *IEEE Transactions on Network and Service Management*.

[6] Shi J., He G., Liu X. Anomaly Detection for Key Performance Indicators through Machine learning.

[7] Jia Z., Lin Y., Liu Y., Jiao Z., Wang J (2020). Refined nonuniform embedding for coupling detection in multivariate time series. *Physical Review*.

[8] Jia Z., Cai X., Hu Y. (2022). Delay propagation network in air transport systems based on refined nonlinear Granger causality. *Transportation Business: Transport Dynamics*.

[9] Yang C., Liu Y., Xiao J., Huang X., Chen J. (2021). Research on intelligent operation and maintenance model of large database for electric power industry. *Journal of Physics: Conference Series*.

[10] Xu Y., Chen N., Huang R., Zhang H KPI data anomaly detection strategy for intelligent operation and maintenance under cloud environment.

[11] Curry D. M., Beaver W. W., Dagli C. H. A System-Of-Systems Approach to Improving Intelligent Predictions and Decisions in a Time-Series environment.

[12] Jia Z., Lin Y., Wang J. (2021). Multi-view spatial-temporal graph convolutional networks with domain generalization for sleep stage classification. *IEEE Transactions on Neural Systems and Rehabilitation Engineering*.

[13] Jia Z., Junyu J., Zhou X. (2022). Hybrid Spiking Neural Network for Sleep EEG Encoding. *Science China Information Sciences*.

[14] Li Z., Wang J., Jia Z., Lin Y. Learning space-time-frequency representation with two-stream attention based 3D network for motor imagery classification.

[15] Jia Z., Cai X., Jiao Z. (2022). Multi-modal physiological signals based squeeze-and-excitation network with domain adversarial learning for sleep staging. *IEEE Sensors Journal*.

[16] Shaterian M., Abrishamifar A., Shamsi H. (2012). Analysis and design of the true piecewise approximation logarithmic amplifiers. *Analog Integrated Circuits and Signal Processing*.

[17] Reasenberg P. (1985). Second-order moment of central California seismicity, 1969-1982. *Journal of Geophysical Research: Solid Earth*.

[18] von Neumann J. (1941). Distribution of the ratio of the mean square successive difference to the variance. *The Annals of Mathematical Statistics*.

[19] Williams B. M., Durvasula P. K., Brown D. E. (1998). Urban freeway traffic flow prediction: application of seasonal autoregressive integrated moving average and exponential smoothing models. *Transportation Research Record: Journal of the Transportation Research Board*.

[20] Gardner E. S. (1985). Exponential smoothing: the state of the art. *Journal of Forecasting*.

[21] Huang J., Li C., Yu J. Resource Prediction Based on Double Exponential Smoothing in Cloud computing.

[22] Belgiu M., Drăguţ L. (2016). Random forest in remote sensing: a review of applications and future directions. *ISPRS Journal of Photogrammetry and Remote Sensing*.

[23] Qi Y. (2012). *Random forest for Bioinformatics, Ensemble machine learning*.

[24] Liu D., Zhao Y., Xu H. Opprentice: Towards Practical and Automatic Anomaly Detection through Machine learning.

[25] Sagi O., Rokach L. (2018). Ensemble learning: a survey. *WIREs Data Mining and Knowledge Discovery*.

[26] Dietterich T. G. (2002). Ensemble learning. *The handbook of brain theory and neural networks*.

